# Omnivore and vegetarians show similar body composition and skin physiology across body regions—A comparative analysis

**DOI:** 10.1111/srt.13798

**Published:** 2024-07-09

**Authors:** Sérgio Fallone de Andrade, Cíntia Ferreira‐Pêgo, Tatiana Fontes, Sofia Lopes, Luís Monteiro Rodrigues

**Affiliations:** ^1^ CBIOS – Research Center for Biosciences & Health Technologies Universidade Lusófona School of Health Sciences Lisbon Portugal

**Keywords:** body composition, diet pattern, omnivore, skin physiology, skin proportional index, vegetarian

## Abstract

**Background:**

Skin physiology seems to be influenced by dietary choices and body composition, although links between these factors remain poorly characterised. In the present manuscript, we elaborate on the potential relationships among food groups, body composition and skin physiology in omnivores and vegetarians.

**Material and Methods:**

This cross‐sectional observational study involved 181 participants, 129 omnivores and 52 vegetarians. The main functions of the skin measured in our laboratory were transepidermal water loss, deep and superficial epidermal hydration, skin elasticity, and carotenoid content. Skin variables obtained from different body regions were made comparable by a new Proportional Skin Index calculated to respect their relative representativity.

**Results:**

No statistical differences were found when comparing both groups' body composition and skin variables from different body regions, with the exception of the skin carotenoid content significantly higher in the vegetarian group (*p* < 0.001).

**Conclusion:**

Although dietary patterns significantly differed between groups, with vegetarians consuming fewer animal‐derived products and more plant‐based foods, multiple linear regression analysis revealed no differences or association between the dietary pattern and the skin physiology. These findings highlight the need for further research to elucidate the specific impact of diet and food groups and body composition on skin physiology.

## 1 INTRODUCTION

The complex equation of factors influencing skin health seems to involve dietary choices and lifestyles,^1^, ^2^ even if related evidence is often dispersed and, in many cases, difficult to obtain. Systematic reviews focused on food nutrition and skin are scarce and insufficient,^3^, ^4^, ^5^, ^6^, ^7^ with only a few studies able establish significant links between these players.^3^, ^4^

Literature has shown a growing body of results relating specific food groups and nutrients in different skin conditions. For example, polyunsaturated fatty acids have been associated with anti‐inflammatory effects and are capable of improving psoriasis and atopic dermatitis.^8^ Fruits and vegetables have long been associated with a protective effect against skin aging and photoaging, attributed to their antioxidant content.^9^, ^10^ On the opposite side, high glycaemic load diets have been related to exacerbated acne.^10^ Only a few current systematic reviews highlighted the importance of nutritional patterns to promote a healthy skin condition and preservation, allegedly influencing skin aging.^6^, ^7^, ^11^

A well‐known and long‐acknowledged difficulty in broad skin studies is related to skin heterogenicity.^12^, ^13^ Epidermis basal layer architecture greatly varies with skin region and also involves hair follicles, eccrine sweat glands and melanocytes, determining different physiological performances that also differ with race and sex, and change during our lifetime as we age. Additional complexities arise from the chemical (molecular) composition of skin related to histology and cell distribution, as well as differences in the microbiome and lifestyles, including daily (hygiene) habits.^14^, ^15^ Thus, it is clear that skin morphology and related immuno‐metabolo‐physiology will be challenging to compare without attending to those specificities. In fact, when assessing principal skin properties in different body regions, such variables as epidermal water balance, biomechanics or pH are collected in very small areas (in most cases < 1 cm^2^). Since an average adult skin approximately corresponds to 2 m^2^ and some 15% of total body mass,^16^, ^17^ the representativity of those measurements should be questioned. This is the (common) practice of longitudinal studies assessing differences among specific populations comparing different regions and different skin proportionalities.^13^, ^15^, ^16^, ^17^ Comparisons are more plausible when the study focuses specific clinical entities, affecting the same equivalent skin regions or clinical outcomes.^18^, ^19^, ^20^, ^21^

The primary objective of our study was to characterize the skin condition of two healthy groups of participants distinguished by their dietary options—omnivores and vegetarians. Here we aimed to compare major indicators of skin physiology and to identify potential relationships between food groups associated with specific dietary patterns, skin function and body composition. Secondarily, we also addressed this skin representativity issue by proposing a new ‘all regions’ cartography index meant to proportionally represent global skin physiological properties.

## 2 MATERIAL AND METHODS

### 2.1 Sample and study design

Our cross‐sectional observational study involved 181 healthy Caucasoid (medium grade phototypes) of both sexes, aged between 34.7 ± 12.2 years old, recruited between January 2022 and February 2023. This sample was divided into two groups according to their self‐reported dietary regimen, in place for at least one year, as omnivore (*n* = 129) and vegetarian (*n* = 52).

Non‐inclusion criteria were being underage, taking any regular medication/supplement, and/or being sick, pregnant, or breastfeeding. All individuals agreed to participate in the study before data collection through informed written consent. Procedures respected all principles of good clinical practice adopted for human research studies, complying with current ethical standards for human research, following the Declaration of Helsinki^23^ and respective amendments. The study was previously approved by the Ethics Committee of the School of Sciences and Health Technologies from *Universidade Lusófona* (EC.ECTS/P05.21).

### 2.2 Characterization data

Information was gathered during a face‐to‐face interview divided into three phases—(1) general characterization of each participant; (2) physical activity classification considering the International Physical Activity Questionnaire—Short Form^24^; and (3) Food Frequency Questionnaire (FFQ) validated for the Portuguese population to identify the dietary intake.^25^ Participants assignment to each group was determined by the FFQ responses. The vegetarian group, which did not consume any type of meat, meat products, or fish, also included a few individuals following vegan dietary practices, which also exclude the consumption of any food produced by animals, including dairy, eggs and honey. The omnivore group involved all participants regularly consuming meat, meat products or fish in their regular food habits.

Body mass was measured by an electronic scale [0.1 kg accuracy], wearing light clothes and no shoes. Height was self‐reported. Body Mass Index (BMI) was then calculated [BMI = Body mass (kg)/height (m)^2^]^26^.

### 2.3 Morphometry (body composition and skin functional assessment)

Body composition measurements were performed after 12 h of fasting and no exercise for 24 h before measurements^27^ via DXA (Lunar Prodigy™ Advance—General Electric Healthcare; Chicago, Illinois, USA). Chosen variables were Visceral Adipose Tissue (VAT) Subcutaneous Adipose Tissue (SAT) and Total Adipose Tissue (TAT).

For skin measurements, participants were allowed to acclimatize to the laboratory conditions (temperature: 22 ± 2°C; relative humidity: 40%−60%) in a comfortably seated position for about 30 min. Participants were required to not apply any cosmetics or toiletries in the testing areas during the 24 h prior to skin assessment.

Measurements took place in several skin regions considering human skin morpho‐functional diversity, from the face (mid‐forehead and mid‐cheek) to the neck base, the hand (dorsum, central) and the leg (antero‐external 10 cm below the knee). These measures corresponded approximately to 21.5% of total body area (Forehead, Cheek, Neck = 5.5%; Hand = 3.0%; Leg = 13.0%). These proportions, shown in Figure 1, were used to calculate one body weighted means—a Proportional Skin Index (PSIx)—for each skin functional variable measured in different regions. Relevant skin variables were obtained by non‐invasive technologies and included transepidermal water loss (TEWL), a direct indicator of the epidermal ‘barrier’, superficial and deep epidermal hydration, elasticity and carotenoid content. TEWL, expressed in g/m^2^/h, was measured using the Tewameter® (Courage + Khazaka electronic GmbH, Cologne, Germany). Epidermal hydration, expressed in arbitrary units (UA's), was measured by the capacitance‐based MoistureMeterEpid SC and Dtec system (Delphin Technologies, Kuopio, Finland).^28^, ^29^ Elasticity, expressed as Ua/Uf, was assessed by the Cutometer® MPA 580 (Courage + Khazaka electronic GmbH).^29^, ^30^ The skin carotenoid content, measured solely in one randomly chosen palm, was assessed using reflectance spectroscopy (Biozoom, Kassel, Germany).^31^

**FIGURE 1:** Skin surface cartography model showing the relative percentage of each body region regarding an adult skin area of approximately 2 m^2^.

### 2.4 Statistical analysis

Results were expressed as mean ± standard deviation (SD) and as relative frequencies (%) for continuous or categorical variables as appropriate. The Student's *t*‐test was used for comparisons between continuous variables, while for categorical variables, the Chi‐square test was chosen whenever variables followed a normal distribution. The association between dietary patterns, food groups and skin parameters was analysed by logistic regression. Multiple linear regression models were performed to assess the relation among different independent variables and skin descriptors. After testing the assumptions for linear regression and collinearity diagnostics, the most common variables in the models—and thus considered as possible predictor variables on skin parameters—identified by this method were dietary pattern (defined as vegetarian or omnivore), biological sex (defined as male or female), age, BMI, TAT, SAT, VAT and smoking status (defined as smoker, former smoker and non‐smoker). Statistical analysis was performed using Jamovi (Version 2.2, the Jamovi Project, Sydney, Australia). The significance level was set at *p* < 0.05.

## 3 RESULTS

Participants were mainly non‐smokers (77.3%) reporting moderate to high physical activity (75.7%). Regarding body composition, no statistical differences were found between omnivore and vegetarian groups involving body mass, BMI, waist circumference and adipose tissue‐related values (Table 1).

**TABLE 1:** General and anthropometric characteristics of included participants according to the dietary pattern.

	Total population (*n* = 181)	Omnivorous (*n* = 129)	Vegetarians (*n* = 52)	*p*‐value
Sex, % (*n*)				
Women	62.7 (116)	67.0 (86)	58.0 (30)	0.257^b^
Men	37.3 (65)	33.0 (43)	42.0 (22)	
Age, years	34.7 ± 12.2	34.7 ± 13.3	34.4 ± 9.1	0.858^a^
Smoking status, % (*n*)				
Non‐smoker	77.3 (140)	76.7 (99)	78.9 (41)	0.784^b^
Former smoker	11.0 (20)	10.9 (14)	11.5 (6)	
Smoker	11.7 (21)	12.4 (16)	9.6 (5)	
Physical activity levels, % (*n*)				
Low	24.3 (44)	24.8 (32)	23.1 (12)	
Moderate	48.6 (88)	51.2 (66)	42.3 (22)	0.293^b^
High	27.1 (49)	24.0 (31)	34.6 (18)	
Body Mass, kg	67.0 ± 15.0	67.2 ± 16.0	66.5 ± 12.1	0.793^a^
Height, m	1.7 ± 0.1	1.7 ± 0.1	1.7 ± 0.1	0.202^a^
BMI, kg/m^2^	23.7 ± 4.7	23.1 ± 5.2	22.1 ± 3.0	0.307^a^
Waist circumference, cm				
Women	76.3 ± 10.9	75.8 ± 12.2	77.6 ± 11.3	0.928^b^
Men	82.4 ± 10.7	83.6 ± 11.0	79.9 ± 9.9	
TAT, cm^3^	2061 ± 1070	2130 ± 1149	1880 ± 8403	0.285^a^
SAT, cm^3^	1409 ± 734	1481 ± 776	1227 ± 597	0.107^a^
VAT, cm^3^	565 ± 516	569 ± 525	554 ± 499	0.869^a^
VAT/SAT ratio	0.42 ± 0.54	0.41 ± 0.58	0.45 ± 0.43	0.651^a^

*Note*: Data expressed as mean ± Standard Deviation (SD) or % (*n*) for continuous variables or categorical variables, respectively. Significance level *p* < 0.05. *p*‐values for group comparisons between omnivores and vegetarians were tested by ^a^student´s *t*‐test or ^b^chi‐squared test.

Abbreviations: BMI, body mass index; SAT, subcutaneous adipose tissue; TAT, total adipose tissue; VAT, visceral adipose tissue.

Regarding skin physiology, no differences in the Proportional Skin Index (PSIx), TEWL, deep or superficial hydration, or elasticity were found (Table 2). Nevertheless, significantly higher TEWL in the leg and lower superficial hydration in the forehead and neck were observed for vegetarians. Statistically significant differences between groups were only observed for the skin carotenoid content, with higher values found in the vegetarian group (Table 2).

**TABLE 2:** Characterization of principal skin physiological functions in different body regions of all participants grouped by their dietary pattern.

	Total population (*n* = 181)	Omnivorous (*n* = 129)	Vegetarians (*n* = 52)	*p*‐value
TEWL				
Forehead	16.79 ± 9.08	16.81 ± 0.88	16.73 ± 0.87	0.960
Cheek	12.27 ± 5.79	11.92 ± 0.49	13.14 ± 0.80	0.192
Hand	10.78 ± 5.68	10.70 ± 0.51	10.98 ± 0.73	0.758
Neck	5.31 ± 4.19	5.15 ± 0.26	5.69 ± 0.87	0.437
Leg	7.25 ± 6.06	6.78 ± 0.54	8.40 ± 0.78	**0.003**
TEWL PSIx	3.16 ± 1.40	3.07 ± 1.38	3.38 ± 1.45	0.176
Deep hydration				
Forehead	43.2 ± 7.9	43.4 ± 0.7	42.8 ± 1.2	0.651
Cheek	41.4 ± 8.3	41.1 ± 0.7	42.4 ± 1.2	0.332
Hand	40.1 ± 7.4	40.1 ± 0.6	40.2 ± 1.1	0.962
Neck	39.2 ± 6.6	39.3 ± 0.6	38.9 ± 0.77	0.699
Leg	33.5 ± 5.8	33.5 ± 0.4	33.6 ± 1.04	0.898
Deep Hydration PSIx	12.8 ± 1.7	12.8 ± 1.5	12.8 ± 2.1	0.923
Superficial hydration				
Forehead	50.1 ± 13.8	51.4 ± 1.2	47.0± 1.8	**0.049**
Cheek	49.1 ± 13.6	49.5 ± 1.2	48.2 ± 1.8	0.547
Hand	35.7 ± 11.1	35.9 ± 1.0	35.1 ± 1.3	0.655
Neck	58.3 ± 13.8	59.6 ± 1.3	55.2 ± 1.7	**0.046**
Leg	33.5 ± 5.8	33.5 ± 0.4	33.6 ± 1.0	0.898
Superficial Hydration PSIx	13.9 ± 2.5	13.9 ± 2.6	13.9 ± 2.3	0.856
Elasticity				
Forehead	0.94 ± 0.07	0.94 ± 0.08	0.95 ± 0.02	0.506
Cheek	0.46 ± 0.03	0.50 ± 0.03	0.38 ± 0.05	0.118
Hand	0.47 ± 0.03	0.49 ± 0.03	0.40 ± 0.05	0.204
Neck	0.44 ± 0.03	0.46 ± 0.04	0.38 ± 0.05	0.292
Leg	0.46 ± 0.04	0.48 ± 0.03	0.40 ± 0.05	0.243
Elasticity PSIx	0.31 ± 0.03	0.30 ± 0.02	0.30 ± 0.05	0.824
Skin carotenoids	5.31 ± 1.32	5.18 ± 1.31	5.61 ± 1.28	**0.047**

*Note*: Data expressed as mean ± Standard Deviation (SD). Significance level *p* < 0.05 (statistically significant values in **bold**). *p*‐values for group comparisons between omnivores and vegetarians were tested by the Student´s *t*‐test. TEWL, transepidermal water loss. Using each variable obtained in those five regions, one Proportional Skin Index (PSIx) was calculated corresponding to a global proportional representation of the measured variable (Forehead, Cheek, Neck = 5.5%; Hand = 3.0%; Leg = 13.0%).

Table 3 contains the multiple linear regression analysis between the dietary pattern and skin parameters. Within the analysed sample, it was not possible to establish an association between dietary patterns (vegetarian or omnivorous) and basic skin physiology represented by TEWL, hydration and biomechanics (*p* > 0.05). Nevertheless, skin carotenoids were statistically associated with a vegetarian dietary pattern (*p* = 0.028). This association remained unchanged after adjustment for different confounders (*p* = 0.021).

**TABLE 3:** Multiple linear regression from (crude and adjusted) data relating dietary pattern and skin variables obtained from different body regions and represented in each case by the respective Proportional Skin Index (PSIx). The carotenoid content was detected in the palm of the hand (see text).

Skin variable	Crude model OR (95% CI)	*p*‐value	Adjusted model OR (95% CI)	*p*‐value
TEWL PSIx	1.15 (0.93–1.44)	0.184	1.11 (0.91–1.37)	0.325
Deep Hydration PSIx	1.01 (0.83–1.23)	0.282	1.05 (0.46–1.15)	0.923
Superficial Hydration PSIx	0.98 (0.70–1.65)	0.855	1.01 (0.93–1.21)	0.458
Elasticity PSIx	0.92 (0.35–1.68)	0.404	0.89 (0.37–1.75)	0.823
Skin carotenoids	1.33 (1.00–1.76)	**0.046**	1.44 (1.02–2.04)	**0.036**

*Notes*: Significance level *p* < 0.05 (statistically significant values in **bold**). Adjusted model for sex, BMI, smoking status, physical activity practice, skin type, and age. The vegetarian group was considered as the reference (REF = 1).

Abbreviations: CI, confidence interval; OR, odds ratio.

Food group consumption significantly differed between both dietary groups, where vegetarians showed a lower consumption of milk and dairy products, meat, fish, eggs, oils, fast food and soft drinks, and a higher daily intake of pulses (Table 4).

**TABLE 4:** Food group consumption according to dietary pattern.

	Total population (n = 181)	Omnivore (*n* = 129)	Vegetarian (*n* = 52)	*p*‐value
Dairy products, g/day	209.0 ± 320.0	287.0 ± 349.0	15.8 ± 50.4	**<0.001**
Vegetable drinks, g/day	98.2 ± 176.0	85.3 ± 157.0	130.0 ± 215.0	0.121
Meat and derivatives, g/day	86.5 ± 167.0	121.0 ± 187.0	0.0 ± 0.0	**<0.001**
Fish, g/day	63.7 ± 75.3	89.4 ± 75.2	0.0 ± 0.0	**<0.001**
Blue Fish, g/day	35.4 ± 41.4	49.7 ± 41.2	0.0 ± 0.0	**<0.001**
Eggs, g/day	35.6 ± 52.9	46.3 ± 58.6	8.9 ± 15.5	**<0.001**
Cereals, derivatives and tubers, g/day	84.1 ± 70.4	86.8 ± 79.2	77.6 ± 41.2	0.433
Pulses, g/day	185.0 ± 130.0	151.0 ± 108.0	267.0 ± 143.0	**<0.001**
Fruits and vegetables, g/day	246.0 ± 176.0	236.0 ± 184.0	273.0 ± 154.0	0.199
Fats and oils, g/day	69.1 ± 38.0	72.9 ± 39.5	59.6 ± 32.3	**0.033**
Fast‐food and soft drinks, g/day	128.0 ± 136.0	146.0 ± 143	83.0 ± 106.0	**0.005**
Fluid intake, L/day	2.0 ± 0.82	2.0 ± 0.71	2.04 ± 1.06	0.467

*Note*: Data expressed as mean ± Standard Deviation (SD). Significance level *p* < 0.05 (values in **bold** type). *p*‐values for group comparisons between omnivore and vegetarians were tested by student´s *t*‐test.

Linear regression allowed us to assess the impact of these different food groups’ consumption on skin physiology, including skin carotenoids (Table 5). Again, no significant differences were observed between groups. Multiple linear regression was further explored, as shown in Table 6. Results suggest that TEWL, deep and superficial hydration, elasticity, and carotenoids do not seem to be influenced directly by adipose tissue (SAT and VAT), waist circumference or BMI.

**TABLE 5:** Multiple linear regression from (crude and adjusted) data relating consumed food by both dietary groups and skin variables.

	TEWL PSIx		Deep hydration PSIx		Superficial hydration PSIx		Elasticity PSIx		Skin carotenoids	
	Crude model OR (95% CI)—(*p*‐value)	Adjusted model OR (95% CI)—(*p*‐value)	Crude model OR (95% CI)—(*p*‐value)	Adjusted model OR (95% CI)—(*p*‐value)	Crude model OR (95% CI)—(*p*‐value)	Adjusted model OR (95% CI)—(*p*‐value)	Crude model OR (95% CI)—(*p*‐value)	Adjusted model OR (95% CI)—(*p*‐value)	Crude model OR (95% CI)—(*p*‐value)	Adjusted model OR (95% CI)—(*p*‐value)
Dairy products, g/day	1.12 (0.31–1.49) (0.337)	1.22 (0.79–1.54) (0.548)	1.08 (0.91–1.28) (0.376)	1.20 (0.89–1.62) (0.211)	1.10 (0.98–1.24) (0.102)	1.08 (0.92–1.27) (0.305)	1.15 (0.55–1.39) (0.823)	1.22 (0.69–1.36) (0.291)	0.91 (0.70–1.18) (0.478)	1.13 (0.80–1.59) (0.486)
Vegetable drinks, g/day	0.95 (0.76–1.19) (0.673)	1.16 (0.58–1.30) (0.662)	0.94 (0.79–1.12) (0.496)	0.98 (0.80–1.19) (0.849)	0.95 (0.85–1.07) (0.449)	0.95 (0.83–1.09) (0.505)	1.15 (0.42–1.65) (0.257)	1.20 (0.61–1.33) (0.589)	1.14 (0.89–1.48) (0.279)	1.14 (0.84–1.56) (0.372)
Meat and derivatives, g/day	1.16 (0.93–1.46) (0.180)	1.22 (0.89–1.67) (0.211)	0.97 (0.81–1.16) (0.765)	0.78 (0.56–1.08) (0.145)	0.98 (0.86–1.11) (0.774)	0.99 (0.85–1.16) (0.961)	1.17 (0.59–1.79) (0.576)	1.19 (0.65–1.41) (0.968)	0.81 (0.62–1.06) (0.133)	0.88 (0.63–1.23) (0.476)
Fish, g/day	0.96 (0.76–1.19) (0.708)	0.97 (0.41–1.29) (0.952)	1.06 (0.89–1.26) (0.504)	1.14 (0.81–1.60) (0.443)	1.06 (0.94–1.20) (0.273)	1.11 (0.94–1.32) (0.194)	1.01 (0.67–1.64) (0.428)	0.99 (0.42–1.33) (0.990)	0.84 (0.65–1.09) (0.194)	0.97 (0.68–1.37) (0.876)
Blue Fish, g/day	1.00 (0.80–1.25) (0.551)	1.04 (0.46–1.37) (0.920)	1.18 (0.98–1.42) (0.091)	1.20 (0.90–1.62) (0.206)	1.05 (0.94–1.19) (0.340)	1.13 (0.96–1.34) (0.139)	1.21 (0.69–1.87) (0.418)	1.16 (0.76–1.65) (0.515)	0.85 (0.65–1.10) (0.215)	1.05 (0.73–1.50) (0.773)
Eggs, g/day	0.96 (0.74–1.25) (0.794)	0.93 (0.68–1.21) (0.934)	1.12 (0.92–1.37) (0.239)	1.08 (0.83–1.39) (0.559)	1.00 (0.88–1.15) (0.930)	0.99 (0.84–1.16) (0.935)	0.99 (0.53–2.01) (0.656)	0.85 (0.38–1.91) (0.710)	1.00 (0.74–1.35) (0.958)	1.12 (0.78–1.59) (0.523)
Cereals, derivatives and tubers, g/day	1.29 (1.01–1.65) (0.122)	1.22 (0.28–1.30) (0.790)	1.02 (0.86–1.22) (0.754)	0.83 (0.66–1.04) (0.107)	0.96 (0.85–1.08) (0.539)	0.94 (0.82–1.08) (0.416)	1.09 (0.77–1.34) (0.739)	1.08 (0.73–1.22) (0.753)	0.93 (0.72–1.20) (0.599)	1.05 (0.78–1.41) (0.738)
Pulses, g/day	1.04 (0.4–1.31) (0.673)	1.05 (0.81–1.36) (0.705)	0.88 (0.73–1.05) (0.160)	0.80 (0.63–1.22) (0.304)	0.91 (0.80–1.02) (0.121)	0.92 (0.80–1.02) (0.265)	0.89 (0.51–1.68) (0.723)	0.83 (0.41–1.65) (0.987)	1.18 (0.92–1.54) (0.184)	1.17 (0.87–1.59) (0.290)
Fruits and vegetables, g/day	0.86 (0.68–1.09) (0.206)	1.21 (0.51–1.96) (0.793)	1.04 (0.87–1.23) (0.648)	1.14 (0.94–1.39) (0.175)	1.04 (0.93–1.18) (0.447)	1.09 (0.95–1.26) (0.181)	1.33 (0.38–2.37) (0.823)	1.13 (0.58–2.17) (0.715)	1.03 (0.80–1.32 (0.809)	0.87 (0.65–1.16) (0.353)
Fats and oils, g/day	1.10 (0.88–1.38) (0.394)	1.29 (0.63–1.77) (0.234)	0.99 (0.84–1.18) (0.942)	0.95 (0.78–1.16) (0.674)	1.02 (0.90–1.15) (0.735)	0.95 (0.83–1.09) (0.515)	1.21 (0.62–1.33) (0.566)	1.21 (0.62–1.33) (0.566)	0.82 (0.64–1.06) (0.140)	0.92 (0.68–1.24) (0.599)
Fast‐food and soft drinks, g/day	1.38 (1.06–1.80) (0.140)	1.25 (0.93–1.68) (0.560)	1.15 (0.96–1.38) (0.112)	1.04 (0.86–1.26) (0.630)	1.06 (0.94–1.19) (0.304)	1.04 (0.90–1.19) (0.578)	1.07 (0.85–1.43) (0.184)	1.03 (0.76–1.82) (0.233)	0.68 (0.51–0.89) (0.111)	0.79 (0.59–1.07) (0.130)
Fluid intake, L/day	1.12 (0.67–1.41) (0.884)	1.09 (0.77–1.33) (0.630)	1.02 (0.78–1.14) (0.216)	0.99 (0.72–1.18) (0.425)	1.05 (0.90–1.18) (0.115)	1.01 (0.91–1.17) (0.358)	1.22 (0.82–1.62) (0.205)	1.18 (1.01–1.51) (0.354)	1.20 (0.92–1.56) (0.162)	1.21 (0.91–1.61) (0.187)

*Note*: Significance level *p* < 0.05. Adjusted model for biological sex, BMI, smoking status, physical activity practice, skin type, age, dietary pattern.

Abbreviations: CI, confidence interval; OR, odds ratio; PSIx, proportional skin index; TEWL, transepidermal water loss.

**TABLE 6:** Multiple linear regression from (crude and adjusted) data relating body composition and skin variables.

	TEWL PSIx		Deep hydration PSIx		Superficial hydration PSIx		Elasticity PSIx		Skin carotenoids	
	Crude model OR (95% CI)—(*p*‐value)	Adjusted model OR (95% CI)—(*p*‐value)	Crude model OR (95% CI)—(*p*‐value)	Adjusted model OR (95% CI)—(*p*‐value)	Crude model OR (95% CI)—(*p*‐value)	Adjusted model OR (95% CI)—(*p*‐value)	Crude model OR (95% CI)—(*p*‐value)	Adjusted model OR (95% CI)—(*p*‐value)	Crude model OR (95% CI)—(*p*‐value)	Adjusted model OR (95% CI)—(*p*‐value)
Fat mass, cm^3^	1.08 (0.87–1.35) (0.448)	1.01 (0.76–1.30) (0.995)	1.16 (0.96–1.41) (0.109)	0.98 (0.77–1.25) (0.913)	1.01 (0.15–1.05) (0.781)	0.83 (0.62–1.11) (0.219)	1.16 (0.51–1.68) (0.362)	1.31 (0.80–1.64) (0.565)	0.92 (0.72–1.19) (0.572)	0.90 (0.68–1.21) (0.508)
SAT, cm^3^	1.06 (0.85–1.32) (0.575)	1.00 (0.77–1.28) (0.969)	1.16 (0.96–1.41) (0.116)	0.99 (0.78–1.25) (0.959)	0.91 (0.90–1.14) (0.781)	0.71 (0.35–1.42) (0.338)	1.21 (0.60–1.41) (0.329)	1.10 (0.56–1.64) (0.958)	1.00 (0.78–1.27) (0.989)	1.09 (0.82–1.45) (0.516)
VAT, cm^3^	0.98 (0.79–1.22) (0.384)	0.90 (0.69–1.16) (0.413)	1.12 (0.95–1.28) (0.202)	1.01 (0.79–1.28) (0.916)	1.08 (0.96–1.22) (0.154)	0.64 (0.32–1.30) (0.227)	1.15 (0.50–1.75) (0.346)	1.21 (0.52–1.44) (0.595)	0.85 (0.67–1.10) (0.223)	0.83 (0.62–1.11) (0.219)
VAT/SAT ratio	0.96 (0.78–1.20) (0.767)	0.99 (0.78–1.26) (0.965)	0.90 (0.74–1.09) (0.298)	0.84 (0.66–1.06) (0.336)	1.04 (0.92–1.17) (0.496)	0.80 (0.41–1.57) (0.523)	1.28 (0.42–1.88) (0.615)	1.27 (0.51–1.91) (0.631)	0.94 (0.73–1.20) (0.621)	0.89 (0.67–1.17) (0.890)
Waist circumference, cm	1.12 (0.90–1.41) (0.307)	1.01 (0.76–1.36) (0.934)	1.15 (0.95–1.39) (0.148)	0.96 (0.76–1.22) (0.767)	0.87 (0.77–0.98) (0.320)	1.04 (0.82–1.33) (0.710)	0.72 (0.44–1.74) (0.808)	1.28 (0.36–1.34) (0.898)	1.21 (0.94–1.55) (0.126)	1.24 (0.93–1.65) (0.137)
BMI, kg/m^2^	1.10 (0.88–1.39) (0.378)	1.09 (0.84–1.41) (0.486)	0.87 (0.69–1.10) (0.258)	0.84 (0.63–1.11) (0.212)	1.00 (0.87–1.15) (0.955)	0.64 (0.29–1.40) (0.268)	1.22 (0.82–1.55) (0.308)	1.19 (0.85–1.67) (0.737)	0.94 (0.71–1.26) (0.712)	0.90 (0.65–1.25) (0.831)

*Note*: Significance level *p* < 0.05. Adjusted model for biological sex, smoking status, physical activity practice, skin type, age, dietary pattern.

Abbreviations: CI, confidence interval; OR, odds ratio; SAT, subcutaneous adipose tissue; TEWL, transepidermal water loss; VAT, visceral adipose tissue.

## 4 DISCUSSION

Vegetarian diet has been referred to improve skin health and appearance when compared to an omnivore diet by favouring barrier function, hydration and elasticity.^2^, ^7^, ^32^ The present manuscript addresses precisely these relationships recognised as major issues in nutrition physiology. Our approach is innovative, as we look deeper into potential relationships amid dietary patterns, food groups, body composition and skin. Further, and importantly, we observe a few experimental details that are often poorly regarded, although crucial for a science‐based judgement. As previously discussed, the diverse composition and functions of the skin are influenced by multiple body determinants and change with race, sex, age and lifestyles. This heterogeneity challenges many studies. The use of single‐point in vivo measurement technologies, involving very small extents that represent only a minor area of this substantial organ, limits the utility of global skin function assessment.

Our data found no differences between the skin of omnivores and vegetarians as expressed by this Proportional Skin Index, a new descriptor here proposed to proportionally describe the same variable obtained in different body sites with different area/volume representativity (Figure 1 and Tables 2, 3, 4, 5, 6). Some statistically significant differences between both groups were found for TEWL measured in the leg, higher in the vegetarian group (*p* < 0.003) and superficial hydration was significantly lower (*p* < 0.05) in the forehead and neck in the same group compared to omnivores (Table 2). The physiological significance of these differences cannot be determined based on the data collected in this study.

Interestingly, skin carotenoid content differences between groups were barely significant (*p* = 0.046). These complex compounds were recently made accessible (non‐invasively) through the skin by spectroscopy. Previous research has demonstrated a direct relationship between these nutrients and lifestyles, including a healthy diet rich in fruit and vegetables.^33^, ^34^ Preliminary studies on carotenoid kinetics demonstrated the sensitivity of these nutrients to stress factors such as sun radiation, environmental hazards or pathophysiological processes.^34^ Currently, it is accepted that a high concentration of carotenoids in the skin provides the best protection strategy against skin photo‐induced aging, especially for lower‐grade phototypes. Recent studies have suggested the interest of vegetarian diets in preserving a good skin condition, mostly related to the high antioxidant properties of the diets.^35^, ^36^ Recently published reviews seem to confirm the wide photoprotection capacities of some of dietary components, carotenoids in particular, and the potential benefits associated with their prevalence in diet.^37^, ^38^ This evidence led us to expect a better physiological performance from vegetarians´  skin compared to omnivores. However, results focused on elasticity, one of the most common descriptors used in human studies,^28^, ^29^ depicted no differences between the two groups (Table 3). By further analysing the potential relationship between the dietary pattern and these skin variables by multiple regression also adjusted for sex, BMI, smoking status and physical activity, significant differences between both groups could only be found for the skin carotenoid content (Table 3).

Significant differences in food consumption emerged, as expected, between omnivorous and vegetarian groups (Table 4). Vegetarian participants showed lower consumption of milk and dairy products, meat, fish, eggs, oils, fast food and soft drinks compared to their omnivorous counterparts. Our results are in line with the current characterization of vegetarian diets, where the prominence of plant‐derived foods is noted alongside the exclusion of practically all animal‐origin products. The consumption of eggs, a nutrient‐rich food source for proteins, including collagen and elastin precursors in particular, were expected to relate positively with skin elasticity.^38^, ^39^ However, no such relationships could be found (Table 5).

Another main nutrient is water. Daily water requirements are still not clearly defined, although a few studies have suggested that a regular diet does not supply all the water needed for daily physiological processes.^39^, ^40^, ^41^ Regarding human skin, a water supplementation study in a healthy omnivore group, adding 2 L/day for 30 days to participants’ regular diets, significantly improved their superficial and deep skin hydration, as well as biomechanical descriptors.^40^ Recent studies confirmed the interest of dietary water in skin homeostasis and relief of dryness, roughness and irritation.^42^ However, no differences in total fluid daily intake between groups or any relationship with skin physiological variables were found (Table 5).

Vegetarian diets have been linked to weight loss, BMI decreases, and fat mass reduction.^36^, ^43^ Our results, however, showed no association between these factors (Table 6), and we note that the mean BMI was similar for both groups (Table 1).

As far as our knowledge goes, our study is the first to look widely into these potential relationships among dietary patterns, body composition, and skin physiology. Although recognizing some limitations, mainly related to (1) the sample dimension and representativity, (2) this relative scarcity of differences and (3) a new skin index not yet validated, we trust the rigor of our approach, supported by a validated FFQ, referenced assessment instruments for quantitative analysis of body functions and composition, and better comparisons of skin dimension.

## 5 CONCLUSION

The skin carotenoid content was the only variable significantly distinct between vegetarian and omnivorous dietary groups. Future research should further explore the specific impact of food groups on specific skin variables, eliminating potential confounding factors to refine and better understand the dynamic interplay between nutrition and skin health and its functional and esthetic preservation.

## CONFLICT OF INTEREST STATEMENT

The authors declare no conflict of interest.

## Data Availability

The data that support the findings of this study are available on request from the corresponding author. The data are not publicly available due to privacy or ethical restrictions.

## References

[1] Tobin DJ . Biochemistry of human skin—our brain on the outside. Chem Soc Rev. 2006;35(1):52–67.16365642 10.1039/b505793k

[2] Boelsma E , Van De Vijver LP , Goldbohm RA , Klöpping‐Ketelaars IA , Hendriks HF , Roza L . Human skin condition and its associations with nutrient concentrations in serum and diet. Am J Clin Nutr. 2003;77(2):348–355.12540393 10.1093/ajcn/77.2.348

[3] Pappas A , Liakou A , Zouboulis CC . Nutrition and skin. Rev Endocr Metab Disord. 2016;17(3):443–448.27401878 10.1007/s11154-016-9374-z

[4] Akalın G , Selamoglu Z . Nutrition and foods for skin health. J Pharm Care [Internet]. 2019 [cited 2024 Feb 20];7(1–2):31–33. https://publish.kne‐publishing.com/index.php/JPC/article/view/1620

[5] Michalak M , Pierzak M , Kręcisz B , Suliga E . Bioactive compounds for skin health: a review. Nutrients. 2021;13(1):203.33445474 10.3390/nu13010203PMC7827176

[6] Leitão C , Mignano A , Estrela M , et al. The effect of nutrition on aging—a systematic review focusing on aging‐related biomarkers. Nutrients. 2022;14(3):554.35276919 10.3390/nu14030554PMC8838212

[7] Cao C , Xiao Z , Wu Y , Ge C . Diet and skin aging—from the perspective of food nutrition. Nutrients. 2020;12(3):870.32213934 10.3390/nu12030870PMC7146365

[8] Ziboh VA , Miller CC , Cho Y . Metabolism of polyunsaturated fatty acids by skin epidermal enzymes: generation of antiinflammatory and antiproliferative metabolites. Am J Clin Nutr. 2000;71(1):361S‐366S.10617998 10.1093/ajcn/71.1.361s

[9] Hughes MCB , Williams GM , Pageon H , Fourtanier A , Green AC . Dietary antioxidant capacity and skin photoaging: a 15‐year longitudinal study. J Invest Dermatol. 2021;141(4):1111‐1118.e2.e2.32682911 10.1016/j.jid.2020.06.026

[10] Melnik B . Diet in acne: further evidence for the role of nutrient signalling in acne pathogenesis—a commentary. Acta Derm Venereol. 2012;92(3):228–231.22419445 10.2340/00015555-1358

[11] Solway J , McBride M , Haq F , Abdul W , Miller R . Diet and dermatology: the role of a whole‐food, plant‐based diet in preventing and reversing skin aging—a review. J Clin Aesthetic Dermatol. 2020;13(5):38–43.PMC738069432802255

[12] Szabo G . The regional anatomy of the human integument with special reference to the distribution of hair follicles, sweat glands and melanocytes. Philos Trans R Soc Lond B Biol Sci. 1967;252(779):447–485.

[13] Von Stebut E , Helbig D . Anatomische und funktionelle Unterschiede der Haut verschiedener Ethnien. Dermatol. 2023;74(2):80–83.10.1007/s00105-022-05100-736607359

[14] Bouslimani A , Porto C , Rath CM , et al. Molecular cartography of the human skin surface in 3D. Proc Natl Acad Sci [Internet]. 2015 [cited 2024 Apr 20];112(17). https://pnas.org/doi/full/10.1073/pnas.1424409112 10.1073/pnas.1424409112PMC441885625825778

[15] Yi F , Yang X‐X , Yang R‐Y , et al. A cross‐sectional study of Chinese women facial skin status with environmental factors and individual lifestyles. Sci Rep. 2022;12(1):18110.36302888 10.1038/s41598-022-23001-6PMC9613773

[16] John AJUK , Galdo FD , Gush R , Worsley PR . An evaluation of mechanical and biophysical skin parameters at different body locations. Skin Res Technol. 2023;29(2):e13292.36823505 10.1111/srt.13292PMC10155800

[17] Dąbrowska AK , Spano F , Derler S , Adlhart C , Spencer ND , Rossi RM . The relationship between skin function, barrier properties, and body‐dependent factors. Skin Res Technol. 2018;24(2):165–174.29057509 10.1111/srt.12424

[18] Katta R , Desai SP . Diet and dermatology: the role of dietary intervention in skin disease. J Clin Aesthetic Dermatol. 2014;7(7):46–51.PMC410635725053983

[19] Katta R , Kramer MJ . Skin and diet: an update on the role of dietary change as a treatment strategy for skin disease. Skin Ther Lett. 2018;23(1):1–5.29357214

[20] Shokeen D . Influence of diet in acne vulgaris and atopic dermatitis. Cutis. 2016;98(3):E28–E29.27814423

[21] Alves E , Gregório J , Baby AR , Rijo P , Rodrigues LM , Rosado C . Homemade kefir consumption improves skin condition—a study conducted in healthy and atopic volunteers. Foods. 2021;10(11):2794.34829075 10.3390/foods10112794PMC8622502

[22] Searle T , Ali FR , Carolides S , Al‐Niaimi F . Rosacea and diet: what is new in 2021? J Clin Aesthetic Dermatol. 2021;14(12):49–54.PMC879449335096255

[23] World Medical Association . World Medical Association Declaration of Helsinki: ethical principles for medical research involving human subjects. JAMA. 2013;310(20):2191.24141714 10.1001/jama.2013.281053

[24] Craig CL , Marshall AL , Sjöström M , et al. International physical activity questionnaire: 12‐country reliability and validity. Med Sci Sports Exerc. 2003;35(8):1381–1395.12900694 10.1249/01.MSS.0000078924.61453.FB

[25] Lopes C , Aro A , Azevedo A , Ramos E , Barros H . Intake and adipose tissue composition of fatty acids and risk of myocardial infarction in a male Portuguese community sample. J Am Diet Assoc. 2007;107(2):276–286.17258965 10.1016/j.jada.2006.11.008

[26] Nuttall FQ . Body mass index: obesity, BMI, and health: a critical review. Nutr Today. 2015;50(3):117–128.27340299 10.1097/NT.0000000000000092PMC4890841

[27] Lopes S , Fontes T , Tavares RG , Rodrigues LM , Ferreira‐Pêgo C . Bioimpedance and dual‐energy x‐ray absorptiometry are not equivalent technologies: comparing fat mass and fat‐free mass. Int J Environ Res Public Health. 2022;19(21):13940.36360820 10.3390/ijerph192113940PMC9657485

[28] Mayrovitz HN , Luis M . Spatial variations in forearm skin tissue dielectric constant: Spatial variations in forearm skin TDC. Skin Res Technol. 2010;16(4):438–443.20923455 10.1111/j.1600-0846.2010.00456.x

[29] Rodrigues LM , Fluhr JW , the EEMCO Group . EEMCO guidance for the in vivo assessment of biomechanical properties of the human skin and its annexes: revisiting instrumentation and test modes. Skin Pharmacol Physiol. 2020;33(1):44–60.31747675 10.1159/000504063

[30] Rosado C , Barbosa R , Fernando R , Antunes F , Rodrigues LM . Study of the effect of epidermal overhydration by occlusion, on the skin biomechanical behaviour assessed in vivo with the systems Cutometer®, Reviscometer® and CutiScan®: Estudo do efeito da sobrehidratação epidérmica por oclusão, sobre o comportamento biomecânico da pele in vivo avaliado com os sistemas Cutometer®, Reviscometer® e CutiScan®. J Biomed Biopharm Res. 2015;12(2):203–213.

[31] Darvin ME , Sterry W , Lademann J , Vergou T . The role of carotenoids in human skin. Molecules. 2011;16(12):10491‐10506.

[32] Rezaković S , Pavlić M , Navratil M , Počanić L , Žužul K , Kostović K . The impact of diet on common skin disorders. J Nutr Ther. 2014;3(3):149–155.

[33] Darvin ME , Fluhr JW , Meinke MC , Zastrow L , Sterry W , Lademann J . Topical beta‐carotene protects against infra‐red‐light–induced free radicals. Exp Dermatol. 2011;20(2):125–129.21255091 10.1111/j.1600-0625.2010.01191.x

[34] Lademann J , Meinke MC , Sterry W , Darvin ME . Carotenoids in human skin: carotenoids in human skin. Exp Dermatol. 2011;20(5):377–382.21366698 10.1111/j.1600-0625.2010.01189.x

[35] Fam VW , Charoenwoodhipong P , Sivamani RK , Holt RR , Keen CL , Hackman RM . Plant‐based foods for skin health: a narrative review. J Acad Nutr Diet. 2022;122(3):614–629.34728412 10.1016/j.jand.2021.10.024

[36] Flores‐Balderas X , Peña‐Peña M , Rada KM , et al. Beneficial effects of plant‐based diets on skin health and inflammatory skin diseases. Nutrients. 2023;15(13):2842.37447169 10.3390/nu15132842PMC10343921

[37] Baswan SM , Klosner AE , Weir C , et al. Role of ingestible carotenoids in skin protection: a review of clinical evidence. Photodermatol Photoimmunol Photomed. 2021;37(6):490–504.33955073 10.1111/phpp.12690

[38] Geng R , Kang S‐G , Huang K , Tong T . Boosting the photoaged skin: the potential role of dietary components. Nutrients. 2021; 13(5):1691. doi:10.3390/nu13051691 34065733 PMC8156873

[39] Schagen SK , Zampeli VA , Makrantonaki E , Zouboulis CC . Discovering the link between nutrition and skin aging. Dermatoendocrinol. 2012;4(3):298–307.23467449 10.4161/derm.22876PMC3583891

[40] Palma ML , Tavares L , Fluhr JW , Bujan MJ , Rodrigues LM . Positive impact of dietary water on *in vivo* epidermal water physiology. Skin Res Technol. 2015;21(4):413–418.26058417 10.1111/srt.12208

[41] Cena H , Calder PC . Defining a healthy diet: evidence for the role of contemporary dietary patterns in health and disease. Nutrients. 2020;12(2):334.32012681 10.3390/nu12020334PMC7071223

[42] Popkin BM , D'Anci KE , Rosenberg IH . Water, hydration, and health: Nutr Rev. 2010;68(8):439–458.20646222 10.1111/j.1753-4887.2010.00304.xPMC2908954

[43] Fontes T , Rodrigues LM , Ferreira‐Pêgo C . Comparison between different groups of vegetarianism and its associations with body composition: a literature review from 2015 to 2021. Nutrients. 2022;14(9):1853.35565820 10.3390/nu14091853PMC9104728

